# Recognition of Factors of Postoperative Complications of Knee Osteoarthritis Patients and Comprehensive Nursing Intervention

**DOI:** 10.1155/2021/1840613

**Published:** 2021-11-23

**Authors:** Ying Dong, Pei Zhang, Lidan Fan

**Affiliations:** Shangqiu Institute of Technology, Shangqiu Henan 476000, China

## Abstract

Knee osteoarthritis (KOA) is a degenerative joint disease characterized by articular cartilage degeneration, cartilage exfoliation, osteophyte formation, and synovitis. It seriously affects the knee joint function and quality of life of patients. Total knee arthroplasty is now the most frequently used therapy for end-stage knee arthritis because it can successfully modify the line of lower extremities, restore knee joint function, alleviate pain, and enhance patients' quality of life; nevertheless, it may cause significant trauma and bleeding. It can easily lead to infection and anemia. In this study, the control group chose total knee arthroplasty and the observation group chose total knee arthroplasty combined with PRP. The results showed that the knee joint function score, visual analog score, blood transfusion, total blood loss, total postoperative drainage, and complications in the observation group were superior to those in the control group. Total knee arthroplasty takes a long time and needs a lot of soft tissue incision, which leads to a lot of blood loss and can cause a variety of complications. Gel has been shown in studies to successfully decrease blood loss during and after total knee arthroplasty, enhance knee joint function recovery, and improve patient quality of life. In this paper, the complications and causes of knee osteoarthritis after total knee arthroplasty were studied. Combined with comprehensive nursing intervention for postoperative recovery, it helps to improve the formation of thrombin and calcium ion, which can effectively reduce blood loss, relieve pain, and promote the recovery of knee joint function. This study analyzed the application of total knee arthroplasty combined with gel in the treatment of knee osteoarthritis.

## 1. Introduction

Degenerative knee osteoarthritis is a common orthopedic disease, with degenerative changes of articular cartilage as the core, characterized by articular cartilage destruction and subchondral bone hyperplasia. Related studies show that the incidence of knee osteoarthritis in the middle-aged and elderly population in China can reach 65%, and with the intensification of the aging trend of the population in our country, the incidence of knee osteoarthritis is gradually increasing [1]. Knee osteoarthritis is the fourth leading cause of knee osteoarthritis in women and the eighth leading cause in men in Europe and the United States, according to an epidemiological study performed by the University of Manchester in the United Kingdom. The most common cause of labour loss is knee osteoarthritis, which affects approximately 50 million people in the United States and forces more than 5% of those affected to retire each year [2]. At present, there are many clinical methods for the treatment of knee osteoarthritis, which are mainly divided into two categories: nonoperative treatment and surgical treatment. Nonoperative treatment is mainly oral nonsteroidal anti-inflammatory drugs, intra-articular injection of drugs, and rehabilitation exercise, while surgical treatment is mainly continuous washing and debridement of knee joint cavity, total knee arthroplasty, knee joint single ankle replacement, and so on. The goal of surgical therapy for degenerative knee osteoarthritis patients is to alleviate pain, enhance joint function, and improve the patients' quality of life.

Arthroscopic debridement is a palliative operation with the characteristics of less trauma and quick recovery. It can relieve the pain caused by meniscus degeneration and tear and postpone the time of artificial knee arthroplasty. Gu et al. [3] used knee arthroscopy to treat elderly patients with degenerative knee osteoarthritis. The results showed that the curative effect of knee arthroscopy was significant, the postoperative recovery was faster, and the quality of life was improved. Knee joint function is less affected. The advantages of arthroscopic debridement include a shorter operation time, less bleeding, less trauma, little impact on patients' joint function, thorough cleaning, and the ability to improve knee joint function and intracavitary effusion after surgery; the disadvantage is that for degenerative knee osteoarthritis patients with obvious varus deformities, arthroscopic surgery can only temporarily relieve some symptoms and cannot be used as an alternative operation. Bone marrow mesenchymal stem cells have low immunogenicity, multidirectional differentiation, and immunomodulatory function, which are often used to reduce inflammatory reaction, immune regulation, and injury repair, with better curative effect and less complications. In Karimpour et al.'s study [4], autologous bone marrow mesenchymal stem cell transplantation in the treatment of patients with knee osteoarthritis has good effect, less complications, and can improve joint function, so it is suitable for the treatment of early knee osteoarthritis. In Kawakami et al.'s study [5], Longbei capsule and bone marrow mesenchymal stem cells were used in the experiment of knee osteoarthritis in rats. The results showed that long turtle capsule combined with bone marrow mesenchymal stem cell transplantation was more effective in repairing knee osteoarthritis. At present, the transplantation of bone marrow mesenchymal stem cells is still in the animal experimental stage, and the clinical trial has not been carried out yet. Autogenous cartilage transplantation is the transplantation of relatively normal articular cartilage from the non-weight-bearing part to the cartilage defect to form a smooth and complete articular surface, which is suitable for the treatment of cartilage defect with an area of less than 9 cm^2^. Klompmaker et al. [6] compared the effectiveness of microfracture and autologous chondrocyte transplantation in the treatment of cartilage abnormalities in the knee. The findings indicated that microfracture had a curative effect comparable to an autogenous cartilage transplant. After the surgery, there was no discernible change in joint mobility, discomfort, or stability [7]. It is considered that matrix-induced autologous chondrocyte transplantation opens up a new idea for repairing articular cartilage defects in osteoarthritis. In patients with degenerative knee osteoarthritis, intra-articular injections of platelet-rich plasma improve tissue repair and ligament and bone regeneration and reduce inflammation. Patients' clinical function and pain score improved substantially following three injections of platelet-rich plasma into the articular cartilage. And platelet-rich plasma intra-articular injection is more effective for relatively young patients and patients with lower grade of knee osteoarthritis [8]. Malik et al. [9] compared the clinical efficacy of intra-articular injection of hyaluronic acid and platelet-rich plasma in the treatment of elderly patients with knee osteoarthritis. Platelet-rich plasma intra-articular injection is a good treatment for mild and moderate elderly patients with knee osteoarthritis, and the effect is better than that of hyaluronic acid intra-articular injection. The disadvantage of intra-articular injection of platelet-rich plasma is that patients need to be injected repeatedly, which can easily lead to infection. Proximal tibial osteotomy is mostly suitable for patients under 65 years old and single compartment knee osteoarthritis. Its advantage is that under the guidance of biomechanical principle, the operation is simple, the operation time is short, and the second-stage knee arthroplasty is still feasible. In Nagamitsu et al.'s study [10], 26 patients with simple medial compartment knee osteoarthritis were treated with proximal tibial osteotomy as shown in Figure 1. After treatment, the pain symptoms and joint function were significantly improved. IL-1, IL-6, and IL-17 levels in individuals were reduced On the one hand, proximal tibial osteotomy may increase the pressure bearing area and create a new stressed articular surface; on the other hand, it can decrease the loading on the medial side, reduce medial cartilage attrition, and therefore eliminate or lessen joint discomfort. Although proximal tibial osteotomy may accomplish the goal of cleansing the joint cavity, the joint incision causes significant stress, and patients' recovery is delayed [11–15]. The main complications are neurovascular injury, osteonecrosis at osteotomy, or delayed union of fracture.

Artificial knee arthroplasty is the main surgical method for the treatment of severe degenerative knee osteoarthritis, and it is the ultimate treatment for patients with knee osteoarthritis [16]. Its main disadvantages are periprosthetic infection, loosening, and periprosthetic fracture, and the cost of revision is relatively expensive, and the curative effect is significantly lower than that of the first replacement [17–19]. The therapeutic effects of arthroscopic surgery and artificial knee arthroplasty on 60 patients with knee osteoarthritis were compared. The results showed that artificial knee arthroplasty was effective in the treatment of knee osteoarthritis [20]. Complications such as poor joint healing and deep vein thrombosis may be reduced. The control group had complete knee arthroplasty, whereas the observation group received total knee arthroplasty with PRP. The results showed that the knee joint function score, visual analog score, blood transfusion, total blood loss, total postoperative drainage, and complications in the observation group were superior to those in the control group. Total knee arthroplasty takes a long time and needs a lot of soft tissue incision, which leads to a lot of blood loss and can cause a variety of complications. PRP gel has been shown in studies to successfully decrease blood loss during and after total knee arthroplasty, enhance knee joint function recovery, and improve patient quality of life. In this paper, the complications and causes of knee osteoarthritis after total knee arthroplasty were studied. Combined with comprehensive nursing intervention for postoperative recovery, it helps to improve the formation of thrombin and calcium ion, which can effectively reduce blood loss, relieve pain, and promote the recovery of knee joint function. This study analyzed the application of total knee arthroplasty combined with PRP in the treatment of knee osteoarthritis.

## 2. Pathogenesis

### 2.1. Disease Process

Knee osteoarthritis (KOA), also known as degenerative osteoarthrosis, knee proliferative arthropathy, knee osteoarthritis, and so on, is a kind of chronic aseptic inflammation with chronic degeneration of knee cartilage as the core, involving synovium, bone, primary band, joint capsule, and other structures of the knee joint. The main clinical symptoms are knee joint pain, swelling, stiffness, limited movement, and even joint deformities. At present, the pathogenesis of KOA is not clear. Most studies believe that human articular cartilage basically belongs to hyaline cartilage, which is composed of cartilage matrix and chondrocytes, of which cartilage matrix accounts for 99%, a certain percentage. It is mostly made up of water, type II collagen, and proteoglycan, and it is important for articular cartilage's biomechanical characteristics [21]. There is a dynamic equilibrium between the production and breakdown of different components of articular cartilage under physiological circumstances. Under the action of mechanical factors (such as the change of mechanical axis of lower extremities, increased joint load, and abnormal joint stability) and biological factors (such as age, sex, heredity, and endocrine), articular cartilage wear or abnormal metabolism of chondrocytes, resulting in the dynamic balance between the synthesis and decomposition of articular cartilage components, is broken [22]. Chondrocytes synthesize and release too many proteolytic enzymes to dissolve the cartilage matrix, type II collagen and proteoglycan decompose more than synthesize, and the elasticity of articular cartilage decreases. When the knee joint is loaded and pressed, articular cartilage loses a large amount of interstitial fluid. At the same time, water permeability rises, and synovial fluid degradation enzymes penetrate into articular cartilage, damaging it and causing articular cartilage degeneration and shedding. When the cartilage falls off to the subchondral bone plate exposure, as shown in Figure 2, under the stimulation of joint movement and other factors, the intramedullary blood vessels and fibrous tissue under the bone surface proliferate and constantly produce new bone (smooth surface such as ivory, called ivory degeneration).

The new bone is prone to microfracture, necrosis, and cystic degeneration under stress. On the other hand, the edge of the joint proliferates excessively to form a thicker cartilage circle, which forms an osteophyte through endochondral ossification. When the osteophyte falls into the joint cavity, it can form articular mice (that is, articular loose body). Joint rats, other particles, and degradation products that fall off into the knee joint can stimulate the synovium to produce interleukin (IL), tumor necrosis factor (TNF), prostaglandin E2, and prostaglandin E2 after contact with the synovium. PGE2, neuropeptides, and other metabolites that exacerbate the illness, such as adiponectin, adipocytokines, and others, are significant material bases for the creation and aggravate the degree in many ways, including stimulating chondrocytes to produce lysozyme. It induces synovial angiogenesis, increases the synthesis of inflammatory factors and matrix metalloproteinases in synovial cells, and further destroys intra-articular homeostasis; the abnormal accumulation of fluid puts the articular cavity in a state of high pressure and stimulates the nerves and blood vessels around the knee joint, thus weakening the regulation ability of the knee joint itself. It can reduce the excitation threshold of pain receptors located in subchondral bone, synovium, periosteum, ligaments, fat pads, and joint capsules, leading to pain sensitization, and can directly activate these pain receptors to produce pain. The occurrence of pain makes the knee joint in a protective position to relieve pain and reduces the range of flexion and extension of the affected limb and reduces the load, resulting in a decrease in activity and fixed contracture, resulting in poor blood circulation and substance metabolism around the knee joint. It will be caused by lack of nutrition and degeneration of cartilage after being not improved for a long time. The number of neuroelectric impulses between neuromuscular synapses decreased, the transport of neurotrophic factors decreased, the catabolism of muscle protein was more than synthesis, and muscle atrophy occurred; fibrosis, joint capsules, and ligaments thickened and shortened, limiting the range of motion of joints even further. These variables contribute to a reduction in knee joint stability and an imbalance in the biomechanical balance of the joint, resulting in an aberrant trajectory of the knee joint and a shift in the instantaneous centre during movement, particularly during weight-bearing exercise. It may exacerbate the breakdown of articular cartilage, creating a vicious cycle that accelerates the disease's progression.

### 2.2. Ladder Therapy

Basic treatment includes patient education, exercise therapy, physical factor therapy (physiotherapy for short), and action support therapy. Basic treatment is also suitable for rehabilitation after arthroscopic debridement, especially exercise therapy. It can maintain and increase the muscle strength of the muscles around the knee joint and the range of motion of the knee joint, increase the stability of the knee joint, and improve the joint function, which is of great significance for postoperative rehabilitation. Drug therapy includes control of symptoms and slow-acting drugs for osteoarthritis. There are many kinds of drugs, which have their own indications, adverse drug reactions, and contraindications. In clinical practise, it is essential to examine the patient's age, sex, BMI, fundamental illnesses, medication allergy history, disease severity, and other factors while selecting suitable medicines, with local topical administration taking precedence. The drug treatment after arthroscopic debridement is basically the same. Osteotomy around the knee joint is one of the most important knee salvage surgeries to correct the lower limb force line and change the knee valgus or valgus state to restore the biomechanical balance of knee joint and then delay or even avoid knee arthroplasty in patients with KOA under CT. As shown in Figure 3, the left position shows an obvious difference than the right one. The common osteotomy around the knee joint includes distal femur osteotomy, proximal tibial osteotomy, biplane osteotomy, and proximal fibular osteotomy. The latter three methods are for the treatment of medial compartment osteoarthritis, and proximal fibula osteotomy is based on the “theory of uneven settlement” around the knee joint. Distal femoral osteotomy is primarily used for the treatment of knee valgus deformity with lateral compartment osteoarthritis. The fibular head is osteotomized in the distal 40-70 mm fibula region, and the fibular head is pulled and sunk in the calf muscle to form a lever with the lateral condyle of the tibia as the fulcrum, thus reducing the force on the medial side of the knee joint and correcting the line of force. Compared with tibial osteotomy and biplane osteotomy, this method has the advantages of simple operation, less trauma, and weight-bearing training on the ground after operation. It is more and more widely used in the treatment of medial compartment osteoarthritis in orthopedics.

### 2.3. Surgical Treatment

KOA arthroscopic debridement, that is, arthroscopic joint exploration and debridement of knee osteoarthritis, was first reported by Magnuson in 1941. The concept and specific operation methods of this procedure are introduced. It is a palliative operation to clean and repair mechanical irritants, joint effusion, and damaged tissue in the knee joint cavity under the condition of endoscope. At present, it is widely used in the diagnosis, research, and treatment of knee joint diseases, which can effectively improve the joint function of mild to moderate KOA patients to a certain extent. Under the condition of arthroscopic visualization, the injury of articular cartilage, meniscus, and anterior and posterior crossband, as well as joint debris and loose body in the articular cavity, can be detected to diagnose the disease and evaluate the severity of the disease. Photography, video recording, and pathological biopsy of the lesion can provide important imaging and pathological data for the follow-up study of the disease. Instruments such as basket forceps, planing knife, and vaporisation rod for radiofrequency surgery may be used to restore the articular surface of cartilage, remove bone spurs that obstruct joint mobility, plane hypertrophic synovium, remove worn and torn menisci during the exploration process, and remove diseased tissue that generates inflammatory mediators, imprisoned meniscus and cartilage, and mechanical factors that induce joint strangulation. Reconstruction of the anterior and posterior cruciate ligament to increase the stability of the knee joint and continuous lavage of the joint cavity with normal saline can remove joint debris and inflammatory mediators to prevent secondary intra-articular tissue wear and pathological changes and remove joint effusion to relieve the pressure inside the joint cavity, so as to achieve the purpose of anti-inflammation, analgesia, relieving symptoms, and delaying the development of the disease.

Arthroscopic debridement achieves the purpose of surgical treatment on the premise of minimizing tissue injury as much as possible. Compared with open surgery, arthroscopic debridement has the advantages of small incision, less local injury, and less interference to the normal structure of knee joint. It is easy to accept by patients and popularise in clinic since the postoperative recovery is fast, there are fewer problems, the surgery is straightforward, and the cost is cheap. Arthroscopic debridement can improve the intra-articular environment to some extent and eliminate the secondary pathogenic factors in the joint, but it has little effect on the extra-articular tissues, such as the muscles around the knee joint, patellar band, and joint capsule, and does not improve the pathological process of the loss of balance in the normal connection of intra-articular bone, cartilage, and cartilage matrix from the source. The operation is still a traumatic and invasive operation. The mechanical stimulation of tissue structure during the operation (such as repeated perfusion and cleaning of articular cavity and tissue and planing of synovium) and postoperative local inflammatory reaction caused by blood coagulation, platelet and macrophage degranulation, and secretion of a variety of cytokines will promote microvascular dilatation, hyperemia, and edema; increase vascular wall permeability; affect the local microcirculation; and then cause intra-articular synovial congestion, hypertrophy, intravascular fluid extravasation to the tissue space, and joint swelling. These abnormally secreted bloody secretions and exudates can also stimulate pain receptors in synovium, ligaments, joint capsules, and other places, causing pain sensitization and pain. Complications such as joint hematocele, intra-articular tissue structure adhesion, and fascia compartment syndrome may occur in extreme instances. These postoperative complications will directly affect and hinder the early recovery of joint function. In addition, through the literature research, it is found that the clinical effective rate of this operation is quite different, and the literature reports that it is 30% and 80%. The reason may be related to the doctor's technical operation, the scope of cleaning and repair, postoperative rehabilitation, and other factors. The postoperative problems of the surgery are exacerbated, the severity is worsened, and the recovery time is clearly extended as a result of these factors, affecting the procedure's curative impact and the patients' prognosis. Therefore, KOA arthroscopic debridement is only an important part of treatment, and it has some limitations, so patients undergoing KOA arthroscopic debridement still need rehabilitation treatment after operation, in order to reduce postoperative complications, speed up the process of postoperative rehabilitation, improve the effect of operation, and finally make patients recover knee joint function as soon as possible and delay the progression of disease.

## 3. Postoperative Treatment

### 3.1. Routine Nursing

Routine nursing includes prevention of joint swelling, relief of pain, observation of distal blood circulation of affected limbs, prevention of postoperative infection and venous thrombosis of lower extremities, and use of crutches or walkers, etc., including drug treatment, physiotherapy, and functional exercise, in order to reduce the occurrence of postoperative complications. The operational limb is usually wrapped with elastic bandage and aseptic dressing following the surgery, and the afflicted knee is cold applied periodically for 24 hours. If there is continuous obvious swelling, the cold compress time can be extended to 72 hours. Attention should be paid to avoid local frostbite, raise the affected limb to reduce joint bleeding and surrounding tissue swelling, and avoid knee joint hematoma. Antibiotics can be used properly before, during, and after operation to prevent infection, and low molecular weight heparin sodium can be used to prevent deep venous thrombosis of lower extremities after operation. The isometric contraction training of ankle pump and quadriceps femoris can be carried out on the same day after operation, straight leg raising and skateboard training can be added on the first day after operation, double crutches or walkers can be used to help walk on the ground on the 2nd-3rd day, and step-by-step load training can be started on the operative limbs 0 percent, 25%, 50%, 75%, and 100% weight-bearing; 4 weeks following surgery, when the operative leg can achieve 100% weight-bearing, remove double crutches or walkers. The elastic bandage may be removed on the third day following surgery, depending on the degree of swelling in the knee joint, and the sutures were removed 10 to 14 days after surgery.

### 3.2. Medication

Drug treatment is classified into oral administration, local topical usage, and articular cavity injection, among other things, based on the various methods of drug delivery. Oral drugs include symptom control drugs and slow-acting drugs for osteoarthritis. There are many kinds of oral drugs, which have their own indications, adverse drug reactions, and contraindications. Risk factors need to be evaluated in clinical application. Considering the patient's age, sex, body mass index, basic diseases, history of drug allergy, degree of symptoms, and economic affordability, the most suitable drugs and the lowest effective dose are selected for treatment. It is not necessary to take them for a long time after the symptoms are controlled. Nonsteroidal anti-inflammatory drug is a traditional anti-inflammatory and analgesic drug that has been used in clinic for many years. It can be used as a first-line drug in the treatment. However, it cannot block the development, knee joint pain is easy to relapse after drug withdrawal compared with traditional NSAIDs, celecoxib and rofecoxib have less interference on gastrointestinal tract, kidney, and platelets, but their anti-inflammatory and analgesic effects are not as good as traditional NSAIDs and are more expensive. The comparison between normal and injury position can be seen in Figure 4. Other studies have reported that inhibitors may increase the risk of heart disease, temporary myocardial ischemia, and stroke. Slow-acting medicines are those that must be administered over a lengthy period of time before they may be effective.

Glucosamine, chondroitin sulphate, and collagen are widely used in clinics to alleviate pain, enhance joint function, and postpone the aging process by increasing the metabolism of articular cartilage, regenerating, and preserving articular cartilage. However, the literature reported that the effects of delaying the course of disease and clinical efficacy are quite different; there is some controversy in the selective use of this kind of drugs. It mainly includes NSAIDs and capsaicin, and there are patches, plasters, gel pastes, and other preparations for clinical choice. Compared with other ways of administration, topical drugs have less side effects (basically no effect on the gastrointestinal tract, liver and kidney function, and cardiovascular system); and are easy to use, especially suitable for elderly patients with mild to moderate pain and for patients with moderate and severe pain; and can be treated with oral drugs. However, it cannot be used in patients with damaged skin and patients who are allergic to drugs.

### 3.3. Physical Factor Therapy

Physiotherapy for short belongs to a kind of physiotherapy, including electrotherapy, phototherapy, ultrasonic therapy, and magnetic therapy; each therapy also contains a number of subitems. Physiotherapy can obviously promote the blood circulation and substance metabolism of the local tissue of the knee joint; relieve pain; eliminate soft tissue swelling by absorbing inflammatory mediators and pain factors; control scar hyperplasia; prevent ligament, joint capsule, and other tissue contracture and adhesion; inhibit joint tissue degeneration; and promote joint tissue repair to improve joint function. Physiotherapy has definite short-term effect, few adverse reactions, and simple operation and can reduce drug dosage, but there is a lack of literature to observe the long-term effect. Low-frequency electrotherapy, which includes direct current therapy, neuromuscular electrical stimulation therapy, induction electrotherapy, and other treatments, uses a current of 1-100 Hz to cure illnesses. Low-frequency electrotherapy is a small current, which has a strong stimulating effect on sensory nerve and motor nerve, causes muscle contraction, promotes tissue blood circulation, relieves edema, and relieves pain. The method of using hypothermia to achieve the purpose of treatment is called cryotherapy. Hypothermia reduces vasoconstriction, vascular permeability, exudation, and edema; reduces sensory and motor nerve excitability and conduction velocity; reduces nerve sensitivity; relieves pain; and reduces muscle tension to relieve spasm. During application, attention should be paid to prevent frostbite due to overcooling and protect the normal skin in the cryotherapy area and the surrounding nontherapeutic area. Cold therapy is widely used after arthroscopic surgery. Ice bag cold compress is usually used as a routine nursing treatment, but there is no unified standard in frequency and time. After treatment, the circumference of the knee joint and the swelling degree of the affected limb were compared between the two groups and the range of motion of knee joint. The results showed that there was no significant difference in the indexes between the two groups, and the therapeutic effect was the same. It was observed that the knee joint swelling reached the maximum at 24 hours after operation, and then, the swelling gradually subsided. Continuous ice application for 24 hours following knee arthroscopy is thought to decrease joint swelling and postoperative wound exudation, allowing functional activity to begin as soon as feasible. Many studies have demonstrated that the loss of muscle strength in the muscles around the knee joint and the restriction of joint activity are strongly linked to the development of the disease, and muscle is an essential extra-articular structural foundation for maintaining the knee joint's stability.

When the decrease of muscle strength and the imbalance of muscle strength of the flexion and extensor group of the knee joint can lead to the decrease of the stability of the knee joint, is results in joint mechanical changes and poor joint surface anastomosis, especially in the weight-bearing activity of the knee joint. The effective contact area of the articular surface of malanastomosis decreased, and the stress of local articular cartilage increased abnormally, which aggravated the injury of knee cartilage. The limitation of joint movement itself is one of the symptoms, and when the activity is limited, the impact on joint activity and blood circulation will also aggravate the disease. Arthroscopic debridement is only aimed at cleaning the pathological tissue in the cavity of the knee joint but has little effect on the muscles, ligaments, and joint capsule around the knee joint. Therefore, muscle strength and range of motion training is particularly important in postoperative rehabilitation. Postoperative muscle strength and joint range of motion training can help to maintain and increase muscle strength, prevent muscle atrophy, improve joint proprioception, increase joint stability and coordination, prevent joint contracture, improve circulation and metabolism, prevent lower extremity deep venous thrombosis, promote the healing of injured tissue, and maximise joint function.

At present, according to whether resistance is applied or not, muscle strength training can be divided into resistance training and nonresistance training, and resistance training can be divided into isometric, isotonic, and isokinetic muscle strength training according to the way of muscle contraction. Nonresistance training can be divided into active exercise and active assist exercise according to the help of external force. The selection of muscle strength training methods should comprehensively consider the current muscle strength level of the affected limb, the basic diseases of the patients, and the purpose of treatment as shown in Figure 5: for those with muscle strength at level 2, choose active assist training and cooperate with electrical stimulation, biofeedback therapy, etc.; if the muscle strength reaches grade 3, it can choose active antigravity training; for those with muscle strength at level 4, it can mainly carry out antiresistance training. Ankle pump training, skateboarding, hamstring muscle contraction, quadriceps contraction, straight leg elevation, and other techniques may be used to avoid muscle atrophy and deep venous thrombosis in the lower legs in patients who have had KOA arthroscopic debridement. In the absence of obvious swelling or infection, resistance muscle strength training can be carried out in order to maintain or increase muscle strength and endurance, protect joints, and delay the development of the disease.

## 4. Experiment and Discussion

### 4.1. Experimental Object

Sixty patients with knee osteoarthritis were randomly divided into two groups. There were 60 patients in the observation group as shown in Figure 6, aged from 62 to 82 years old, with an average of 65.71 ± 2.79 years. The average body weight of the patients was 42-82 kg (62.51 ± 2.02 kg). There were 8 cases of diabetes, 11 cases of hypertension, 10 cases of osteoporosis, 6 cases of primary school education, 8 cases of junior middle school, 10 cases of senior high school, and 6 cases above senior high school. There were 22 males and 8 females. There were 19 cases on the left side and 11 cases on the right side, and the course of disease ranged from 13 to 33 months, with an average of 23.12 ± 8.34 months. There were 30 patients in the control group, aged from 62 to 81 years old, with an average of 65.71 ± 2.79 years. The average body weight of the patients was 42-82 kg (62.51 ± 2.02 kg). There were 8 cases of diabetes, 11 cases of hypertension, 10 cases of osteoporosis, 6 cases of primary school education, 8 cases of junior middle school, 10 cases of senior high school, and 6 cases above senior high school. There were 21 men and 9 women in the group. The illness course varied from 13 to 33 months, with an average of 23.15 ± 8.92 months. There were 18 instances on the left side and 12 cases on the right side, and the disease course ranged from 13 to 33 months. Both sets of broad information are similar. The control group chose total knee arthroplasty and routine general anesthesia, adopted anterior median knee incision via medial patellar approach to perform total knee arthroplasty, selected appropriate prosthesis placement and fixation, and carried out rehabilitation exercise after operation. In the observation group, total knee arthroplasty combined with PRP was selected. On the basis of the control group, 60 ml of elbow venous blood was drawn with a preinstalled 8 ml glucose citrate syringe under aseptic condition and shaken well, and the supernatant was selected. The control group was only sprayed with the same amount of normal saline mixed with hemagglutinin. After spraying, the drainage tube is placed and the incision is closed layer by layer.

### 4.2. Experimental Results

After the first treatment of the two groups of patients, compared with the visual analogue scale(VAS) pain score before the implementation of the scheme, the VAS pain score of the two groups decreased significantly after the first treatment, and there was a significant difference, indicating that the two schemes have an immediate effect on joint pain in patients with degenerative knee osteoarthritis. After the first treatment, the comparison between the two groups showed that there was a significant difference in the VAS score between the two groups after the first treatment. Among them, the decrease of VAS pain score in the floating acupuncture group was significantly lower than that in the routine acupuncture group, which revealed that the immediate analgesic effect of floating acupuncture was more significant. After the first treatment, there was a significant difference in recovery rates between the four groups, with the average duration of floating acupuncture being significantly longer than that of routine acupuncture, indicating that floating acupuncture therapy had a significant curative effect, as shown in Figure 7. One month after the end of the regimen, the VAS pain score and scale scores were followed up for both groups of patients, and compared with those before the beginning of the regimen and after treatment, there were significant differences between the two groups. The follow-up scores of the two groups were compared between the two groups, and the mean values of the two groups showed significant differences.

Among them, the average VAS score in the floating acupuncture group showed a curvilinear downward trend at each time point, whereas the average VAS score in the routine acupuncture group was larger than after treatment, but significantly lower than before treatment, while the scale scores in both groups decreased significantly during follow-up and increased compared to those after treatment, but the average increase in the floating acupuncture group was higher than the average increase in the routine acupuncture group. The results show that the two treatment schemes have the persistence of the curative effect, but the curative effect of the routine acupuncture group on knee pain and clinical symptoms of KOA patients is significantly worse than that of the floating acupuncture therapy, and the floating acupuncture therapy has a better continuous therapeutic effect. Pain is the most prominent symptom in patients with degenerative knee osteoarthritis. In the whole course of the development of KOA, pain can change with the gradual evolution of the disease. After receiving certain analgesia treatment, pain symptoms can be effectively relieved, so this study chose the degree of pain as the evaluation index.

Pain is the self-feeling of people's brain after adverse external stimulation, which is a subjective factor, and there is no instrument that can be measured objectively in the current scientific and technological means. The degree of pain is currently mainly quantified by a variety of related pain scales, and among these scales, the VAS pain score should be the most widely used in clinic, and there are many clinical studies using VAS to observe changes in KOA pain, so this clinical study uses VAS to evaluate the changes in knee joint pain. The most prominent symptom of KOA is periarticular pain. At present, the medical community believes that the pain symptoms are caused by inflammatory factors, endocrine, free radicals, basic metalloproteinases, chondrocyte apoptosis, increased intraosseous pressure, and other factors. Among them, the influence of inflammatory factors is the primary mainstream thought at present. For many representatives of the inflammatory cytokine group, the greatest importance is attributed to IL-l, P-force, tumor necrosis factor, IL IL-15, IL-17, and IL-18. The presence of inflammatory cytokines in the joint mainly has a destructive effect on articular cartilage. This is a multilevel impact that causes chondrocytes to age and apoptose, decreases chondrocyte production (such as proteoglycan and II collagen), and directs autoimmune cells to inflamed areas. Among these factors, the increase of intraosseous pressure cannot be ignored; it is closely related to inflammatory factors. When the intraosseous pressure increases, the final result will lead to the gradual increase of inflammatory factors in the joint, which leads to inflammation.

These experiments show that when pressure rises to 5.3 kpa or above, patients will have rest pain around the knee joint, but when IOP is less than 4.7 kpa, there will be no corresponding resting pain, but two cases will occur at the critical point of 3.7 kpa, and knee joint pain will occur occasionally when it is more than 3.7 kpa. The experiment also clearly pointed out that the internal bone of patients with rest pain was basically in a state of high pressure, and the position basically had 40 mmHg as shown in Figure 8. The causes include blood vessels, muscles, and blood flow, among which muscle factors are the most obvious. When the muscles around the joint, such as quadriceps femoris, are contracted by current stimulation, the IOP in the joint can instantly rise to 42 ± 1.1 mmHg. It may revert to its usual range once the stimulus is turned off. Quadriceps femoris contracts, and the blood arteries around it are compressed simultaneously, accelerating arterial blood flow while delaying venous blood flow. This results in intraosseous venous reflux being stagnant and then increasing, as described above. That is exactly how intraosseous venous reflux and stagnation work, according to KOA's primary process of development. The expression function between osteoblasts and osteoclasts is currently out of balance due to the regulation of various biological cytokines, resulting in an imbalance in the bone resorption and reconstruction process, as well as damage to the trabecular bone under cartilage and the bone plate under cartilage. There was an upward trend in the concussion ability produced by local absorption activity as necrotic trabeculae enhanced subchondral bone sclerosis in a gradient, and a downward trend in this process rendered the force on the cartilage contact area unequal. This increased the equivalent pressure on the joint, causing additional cartilage injury.

## 5. Conclusion

Knee osteoarthritis is a disease with joint pain, which can directly affect the patient's movement ability, restrict their movement, and further cause negative psychological problems. Clinical treatment methods are mainly divided into two categories: nonsurgical treatment and surgical treatment. To prevent the occurrence and development of postoperative complications, it is necessary to pay attention to the routine postoperative care of patients, including prevention of joint swelling, pain relief, bandaging, anti-infection, rehabilitation care, and develop personalized plans to prevent postoperative complications. All these can improve the recovery effect of patients after surgery and improve their quality of life.

## Figures and Tables

**Figure 1:** The recovery process of artificial knee arthroplasty.

**Figure 2:** The stimulation of joint movement and other factors.

**Figure 3:** The CT imaging of the left and right injury position.

**Figure 4:** The comparison between normal and injury position.

**Figure 5:** The healing index changes with the healing time.

**Figure 6:** The classification of gonitis patients.

**Figure 7:** The comparison of recovery rates.

**Figure 8:** The determination of the injury position compared to the CT scan.

## Data Availability

The data used to support the findings of this study are included within the article.
